# Is Resilient Transportation Infrastructure Low-Carbon? Evidence from High-Speed Railway Projects in China

**DOI:** 10.1155/2022/3138413

**Published:** 2022-04-28

**Authors:** Zheng He, Genda Wang, Huihua Chen, Hongyan Yan

**Affiliations:** ^1^Central South University, Shaoshan Rd, Railway Campus, Changsha 410075, Hunan, China; ^2^Hunan University of Finance and Economics, Fenglin Rd, Changsha 410205, Hunan, China

## Abstract

Establishing resilient transport infrastructure is an effective way for cities to deal with external disturbances and uncertainties during rapid urbanization. However, human society is presently facing a series of sustainable development obstacles, where the energy shortage and environmental pollution are catching significant concerns. Hence, it is imperative to investigate the carbon emission of the growing number of resilient transportation infrastructure (RTI) projects. Through extracting the carbon emission factor (CEF), this study built the carbon emission measurement model (CEMM) to evaluate the carbon emission of 26 resilient high-speed railway construction projects in China. The results indicated that the carbon emissions of the entire high-speed railway infrastructure projects in China show regional and social environmental differences. Meanwhile, there are potential correlations and positive relationships between the resilience of the high-speed railway infrastructure projects and their carbon emission. Suggestions and recommendations for governments and construction enterprises are put forward to further improve the resilient and low-carbon development of transportation infrastructure in China.

## 1. Introduction

In the past decade, China is undergoing a rapid urbanization process with a high increasing rate of 1.46%. Under this background, a large number of people have poured into the megacities and the capitals of the provinces of China, such as Beijing, Shanghai, Guangzhou, and so on. To effectively alleviate the pressures on the urban caused by the concentration of the large populations, these cities are promoting and improving infrastructure construction. However, the construction projects of urban transport infrastructure, which are served as the lifeline, are challenged by a series of natural or man-made disasters, such as the natural hazards of hurricanes, fires, earthquakes, public security problems, and so on. These disasters act as the most significant uncertainties and disturbances that bring severe damage to the infrastructure, which thus will result in huge economic and social losses for the urban residents [1].

The concept of “resilience,” which owns the unique advantages of the traditional disaster management framework, is one of the efforts made to overcome the challenges [2]. A resilient transport infrastructure with the characteristic of absorption, adaptation, recovery, and upgrading can withstand the external uncertainties and disturbances and maintain the basic function and performance, which finally guarantee the lives and property safety of the residents.

However, the urban transport infrastructure that required huge investments is of both high energy and resource consumption. Can the resilient transport infrastructure meet the current requirements for low-carbon emission? In 2018, global carbon emissions reached the historic high record of 33 billion tons, an increase of 1.7% over the last year [3]. At the same time, China's carbon emissions reached 9.5 billion tons, an increase of 2.5%, accounting for about 28% of the world [4]. China became the country with the largest carbon dioxide emissions in the world, and it is the key area for carbon emission reduction and low-carbon development. Thereafter, China has implemented a series of national strategies to actively respond to climate change achieve low-carbon and sustainable development and promote carbon emission reduction in infrastructure construction [5]. At the end of 2019, China's carbon emissions have been reduced by about 48.1% compared with 2015, reversing the rapid growth of carbon dioxide emissions. In 2021, China aims to “strive to achieve carbon peaks by 2030 and carbon neutrality by 2060.” The “14th Five-Year Plan” has also made comprehensive arrangements for achieving carbon peaking, carbon neutrality, and addressing climate change [6, 7].

On these bases, the resilient transport infrastructure and the low carbon emission share the crucial strategic goals that both are expected to enhance the performance of the city, maintain the steady of the city system, reduce losses bring benefits, and improve the life quality of the residents. Hence, when the transport infrastructure is designed to be resilient, it must also be planned to meet the needs of low carbon emissions.

However, scarce prior studies have investigated the connections between resilient transport infrastructure and low carbon emission. The existed literature focused on making an independent discussion of the resilient transport infrastructure and the low carbon emission separately. Hence, this study aims to investigate the relationship between resilient transport infrastructure and low carbon emissions from this perspective. The tasks of this study are as follows.

## 2. Literature Review

### 2.1. Transport Infrastructure Resilience

The infrastructure is acknowledged as the most critical lifeline of the cities [8–10] which is of great significance for the flow of commerce, city residents, goods and information, and even the daily activities of society [11]. Infrastructure can be considered to include everything from the physical infrastructure of roads, bridges, airports, rail, water supply, telecommunications, and energy services to the social infrastructure of health care, education, banking, and financial services, emergency services, and the justice system [12–15].

The main responsibility of the department of traffic management is to give priority to ensuring that the physical engineering of the transportation infrastructure is intact and that the social services provided by the transportation infrastructure can operate continuously, stably, and safely [16–19]. Compared with traditional risk defensive measures, this demand for the transportation infrastructure system level will attract special attention from the decision-makers and the researchers [20, 21]. Therefore, the resilience proposal helps define, measure, and improve the traditional paradigm in the entire transportation system [22, 23].

From the perspective of the function of the transportation infrastructure construction project, the social and urban producing activities depend on the availability of the transportation network [24–27]. When the transportation infrastructure project operates under uncertain conditions and disturbances and the ability to quickly restore an acceptable level of service after a disruptive event occurs, it is the basis for the survival of the whole city [28, 29].

### 2.2. Carbon Emission

#### 2.2.1. Greenhouse Gas and Environmental Problems

With the progress of human civilization, production activities have become increasingly frequent. Large-scale industrialization activities require the consumption of a large number of fossil fuels, resulting in a large number of cumulative emissions of carbon dioxide [30]. The global accumulation of large amounts of carbon dioxide emissions will cause the concentration of greenhouse gases in the Earth's atmosphere to increase rapidly and significantly, eventually causing a series of environmental problems such as global warming and rising sea levels [31, 32].

These environmental problems will have a significant negative impact on the global natural ecosystem. In addition to global temperature rise and sea-level rise, extreme climate events are also typical climate disaster events, posing a huge threat to human survival and development [33].

The generally accepted view in theoretical circles is that carbon dioxide (CO_2_) is the main greenhouse gas (GHG). If carbon dioxide emissions cannot be controlled and active and effective actions are taken, a series of environmental problems caused by the global climate will bring huge losses to the global economy (about 5% of global GDP each year). Therefore, achieving carbon emission reduction should be the consensus and top priority of everyone.

#### 2.2.2. Carbon Emissions

Carbon emissions refer to the average greenhouse gas emissions produced by byproducts during the life cycle of production, transportation, use, and recycling [34, 35]. In actual research, the total amount of carbon emissions in a certain area can be measured in a certain period. Carbon footprint is usually used to measure the total amount of greenhouse gases released by an organization or product each year. Carbon efficiency is used to quantify carbon footprint efficiency. It is the ratio of carbon dioxide emissions to the company's annual revenue [36, 37].

#### 2.2.3. Carbon Emissions Factor

Carbon emission factor (CEF) refers to the number of carbon emissions produced per unit of energy during combustion or use. The IPCC believes that the carbon emission factor of a certain energy source is fixed. But, every year, the Chinese government announces the carbon emission factors for the six major regions of China.

#### 2.2.4. Carbon Emission Intensity

Carbon emission intensity (CEI) aims to reveal the internal relationship between the level of economic development and carbon emissions in different countries and regions. Its calculation formula is the ratio of carbon emissions to GDP, that is, carbon emission intensity is inversely proportional to GDP. High carbon emission intensity indicates carbon emissions in the region. High energy consumption or low GDP value and low carbon emission intensity indicate that the region's energy use efficiency is high. Per capita, carbon emission is the ratio of the total carbon emissions of a country or region to the population of the region. Per capita, carbon emission can generally measure the level of development of a country or region.

#### 2.2.5. Carbon Emission Measurement Method

Based on applicable objects and measurement scales, carbon emission measurement methods can be divided into four types: field measurement method, carbon emission coefficient method, input-output method, and material balance algorithm [38].

The site measurement method is the most accurate carbon emission measurement method, and its measurement objects are specific and specific carbon emission units [39]. The site measurement method requires the use of specific professional equipment to monitor the emission flow rate and speed of the research gas and then calculate the output carbon emissions. The site measurement method is generally applied to the carbon emission measurement of the ecosystem, and the industrial carbon emission measurement is less used.

The carbon emission coefficient method, also known as the IPCC inventory method, was first proposed by the IPCC (United Nations Intergovernmental Panel on Climate Change). It refers to the establishment of a carbon emission factor database containing all emission units, combing the carbon emission inventory, and obtaining the carbon emission units of activities or products [40]. Multiply the carbon emission unit data on the carbon emission inventory with the corresponding carbon emission factor to obtain the carbon emission of the emission unit and sum them up to obtain the total carbon emission of the research object. This method is similar to the domestic railway engineering quantity inventory pricing method, and the key to its use is to accurately calibrate the carbon emission factor. Many experts and scholars worldwide have calculated and analyzed the carbon emission coefficients of various energy and materials and constructed a rich database of carbon emission factors. Due to the simple calculation logic, strong operability, and relatively easy acquisition of carbon emission data, the carbon emission coefficient method has become the most widely used carbon emission measurement method [41].

The material balance algorithm, also known as the material balance method or the mass balance method, is a method of measuring the material consumption of the research object according to the law of conservation of mass [42]. Material balance refers to the principle of conservation of quality or “four-pillar inventory” in the system per unit time, that is, the original amount of material + the amount of new material = the amount of material consumption + the remaining amount of material. In the actual industrial production process, the use of this method requires first determining the process flow, to obtain the internal connection between the raw materials and the product [43, 44]. The products include the final product, the semi-finished product that has not been processed, and the byproducts produced together with the main product. It is necessary to comprehensively control the material consumption, physical and chemical reactions, and the impact of the environment on the production of products in each production stage and finally analyze and calculate carbon emissions. Because this method needs to master the physical and chemical reactions and energy consumption in each production stage, the calculation logic is complicated and involves a lot of content, and the measurement workload is relatively large.

The input-output method is different from the first three measurement methods. It uses the macro input-output table data to build a model; analyzes the internal connections between different industries, different economic sectors, and macroeconomic data; and combines them to reflect the characteristics of the industry [45]. The environmental impact data of the company estimate the environmental impact of a product. The input-output method has low requirements on the data accuracy and data range of the research object. Using the input-output method does not need to spend a lot of time and energy sorting out the carbon emission inventory. As long as the macro input-output table data are used, the environmental impact of a product can be determined for quick evaluation [46]. In summary, the input-output method is a macroevaluation method that analyzes the overall environmental impact of a certain industry or department and cannot accurately measure the carbon emissions of specific products or objects [47].

#### 2.2.6. Carbon Emission Factor Calibration Method

The key to using the carbon emission coefficient method is to accurately calibrate the carbon emission factor. There are currently the following three mainstream carbon emission factor calibration methods:

1. The carbon emission factor is calibrated based on the equivalent carbon dioxide value produced per unit of energy. This law applies to the calibration of energy carbon emission factors. For example, the carbon emission factors of fossil energy and electricity can be calibrated with the amount of fossil energy consumed per unit mass (volume) and the carbon dioxide emissions produced by consuming 1 kWh of electricity;
2. The carbon emission factor is calibrated based on the equivalent carbon dioxide value produced by the production unit product. This method is applicable to the calibration of carbon emission factors of materials and construction machinery. According to the production process, the carbon dioxide emissions produced by the production unit materials and equipment are measured to achieve the purpose of carbon emission factor calibration;
3. The carbon emission factor is calibrated based on the equivalent carbon dioxide value produced by the direct carbon source consumed. This method is suitable for direct carbon source carbon emission factor calibration. For example, coal can be used to measure the amount of carbon dioxide, nitrogen oxide, and other gases produced after full combustion based on the element composition to achieve carbon emission factor calibration.

This study uses the first two methods to calibrate the carbon emission factor.

## 3. Methodology

As mentioned above, there are many carbon emission measurement methods, and multiple methods are used for accurate measurement in many studies. Since the carbon emission coefficient method has obvious advantages in carbon emission measurement in the fields of construction and engineering, this study chooses the carbon emission coefficient method as the carbon emission measurement method. The carbon emission coefficient method is adapted in this study as the carbon emission measurement method.

### 3.1. Defining the Boundary of Carbon Emission Measurement

The determination of the carbon emission measurement boundary is the first step in the construction of the carbon emission measurement model. The definition of the measurement boundary is subjective, and its breadth and depth directly determine the accuracy and difficulty of carbon emission measurement.

Railway engineering can generally be divided into eight subsystems of bridges and culverts, tunnels, subgrades, tracks, traction power supply, electricity, signal, and communication (the latter four systems are generally collectively referred to as the four-electric system). This paper takes all subsystems into the carbon emission measurement. Meanwhile, we select the “bid section Y of railway X” as the studied cases. However, due to the large amount of railway construction projects and many majors involved, it is difficult to consider all aspects. Therefore, this article only measures the carbon emissions of major energy sources, materials, machinery, and equipment. The carbon emissions of energy, materials, and machinery that do not account for a large proportion are no longer considered. The specific selection criteria are as follows:

1. Quality standards: Classify all building materials consumed in railway construction and sort all types of materials from large to small according to their quality. Materials whose cumulative mass exceeds 80% of the total mass of the materials are included in the measurement range.
2. Cost standard: Classify all materials consumed in railway construction and sort all kinds of materials according to cost from largest to smallest. Building materials whose cumulative cost exceeds 80% of the total material cost are included in the measurement range.
3. Carbon emission standards: Classify all machinery and equipment used in railway construction and sort all types of machinery according to carbon emissions from largest to smallest. Machinery and equipment with cumulative carbon emissions exceeding 80% of the total carbon emissions are included in the measurement scope.

### 3.2. Source of Data

The railway construction process involves a large amount of energy consumption, the use of materials and construction equipment, and a large amount of relevant data is generated, which causes the railway construction carbon emission measurement to rely heavily on data, and the accuracy of the data directly affects the accuracy of the carbon emission measurement results. This study divides the carbon emission measurement data into two major categories: railway engineering quantity data and carbon emission factor data, and explains their data sources and selection methods.

#### 3.2.1. Railway Engineering Volume

Railway engineering volume data is the basis of railway construction carbon emission measurement. Railway engineering volume data mainly includes two parts.

1. Railway construction materials and construction equipment data
2. Railway construction materials and construction equipment data include the types and consumption of construction materials, the types of construction equipment and the number of mechanical shifts, and the energy consumption per mechanical shift. As a large amount of data is involved in the process of railway construction, data accuracy and data availability are considered comprehensively when selecting.
3. The data sources of materials and construction equipment include railway project budget documents, cost software such as Glodon, and engineering drawings. Budget documents generally refer to construction quotas or budget quotas; the built-in quota data in the cost software depend on the productivity levels of different regions, and there may be differences in consumption of the same equipment or process.
4. Railway construction material transportation data
5. The carbon emission generated by the energy consumption during the transportation of a large number of building materials is an important part of the carbon emission of railway construction. The transportation objects in the transportation stage include the building materials, prefabricated components that constitute the railway engineering entity, and turnover materials used in amortization during the construction stage. In the construction material transportation stage, carbon emission measurement should collect data such as the transportation distance, transportation weight, and transportation method of the building materials.
6. It is generally believed that the transportation process includes three parts: one is the raw material mining place to the raw material processing place. The carbon emission factor for building materials calibrated in this paper considers the transportation process of raw materials from the mining place to the processing place, so it is no longer considered in the transportation data. The second is the construction material production site (raw material processing site) to the construction site. This transportation process includes the transportation of turnover materials and prefabricated components used in railway construction. The third is the waste from the construction site to the landfill. The railway construction phase involves the transportation of a large number of wastes such as tunnel slag and abandoned formwork.

In summary, the transportation data in this study need to consider the transportation process of building materials production site (raw material processing site) to a construction site and waste from the construction site to the landfill.

#### 3.2.2. Identification of the Carbon Emission Factor

Carbon emission factor calibration is the core part of carbon emission measurement using the carbon emission coefficient method. Accurate carbon emission factors are the key to achieving accurate carbon emission measurement. The carbon emission factors are identified from the literature (Table 1).

### 3.3. Calibration of the Carbon Emission Factor

Carbon emission factor calibration is the core part of carbon emission measurement using the carbon emission coefficient method. Accurate carbon emission factors are the key to achieving accurate carbon emission measurement. This research sorts out the carbon emission factors of energy, transportation, building materials, and construction machinery and establishes a reliable carbon emission factor database.

#### 3.3.1. Energy CEF

In the railway construction stage, direct consumption of energy or indirect consumption of energy through machinery produces a large number of carbon emissions. Energy carbon emission factors are the basis for the calculation of carbon emission factors for building materials and machinery, so it needs to be clarified first. This article divides energy into fossil energy, electricity, and water.

(1) Fossil energy CEF
Regarding the hot issue of carbon emissions, many institutions actively participate in the research and calculate and publish carbon emission factor data. Among them, the IPCC (United Nations Intergovernmental Panel on Climate Change), as a climate change assessment agency with international influence, published assessment reports five times in 1990, 1995, 2001, 2007, and 2013 and issued research systems, computing science, and comprehensive energy carbon emission factor data. However, since the IPCC's latest assessment report was released in 2013 (IPCC WGI Fifth Assessment Report), the timeliness is poor, and the energy carbon emission factor in the IPCC assessment report is determined based on international data, which is different from China's carbon emission data. Therefore, this cultural stone energy carbon emission factor data does not directly quote the relevant data in the IPCC assessment report but draws on the calculation method of the IPCC energy carbon emission factor and calculates it by China's national conditions. Since the carbon emissions of fossil energy mainly come from the use (consumption) stage and the carbon emissions in the production and transportation stage are difficult to measure, this article only measures the carbon emissions generated during the use (consumption) stage.
According to the benchmark method published in the energy section of the 2006 IPCC National Greenhouse Gas Inventory Guidelines 2019 Revised Edition, the calculation formula for the carbon emission factor of this cultural stone energy (combustion) is
  (1) $$\begin{array}{c} \text{Fossil energy CEF}=\text{default net calorific value}\times \text{default carbon content}\times \text{default carbon oxide factor}\times \text{molar conversion coefficient of carbon and carbon dioxide.} \end{array}$$
In the formula, the default net calorific value is derived from the “China Energy Statistical Yearbook 2018”; the default carbon content is quoted from the “2006 IPCC National Greenhouse Gas Inventory Guidelines 2019 Revised Edition”; the default carbon oxidation factor is 100% (the degree of carbon oxide combustion does not affect its carbon content); the molar conversion coefficient of carbon and carbon dioxide is 44/12. The calculation results of fossil energy carbon emission factors are shown in Table 2.
(2) Electricity CEF
As clean energy, electricity does not directly produce carbon emissions during its use but consumes energy to produce carbon emissions during its production process. Therefore, the carbon emission factor of electricity is affected by the energy structure of power generation. The Climate Change Department of the National Development and Reform Commission has clarified two types of marginal emission factors, OM (marginal emission factor for electricity) and BM (marginal emission factor for capacity) in the “2019 China Regional Grid Baseline Emission Factors,” and unifies the grid boundaries. It is divided into regional power grids in North China, Northeast China, Northwest China, East China, Central China, and South China, excluding Tibet Autonomous Region, Taiwan Province, Hong Kong, and Macau Special Administrative Regions. The carbon emission factors of power in each region are shown in Table 3.
(3) Water CEF
Water does not contain carbon elements, so water is not a direct carbon emission unit but indirectly produces carbon emissions during its production and transportation. Therefore, its carbon emission factor refers to the energy consumption per unit volume (mass) of water production and transportation. Carbon emissions are generated. This study quotes the value of 0.91 kg CO_2_/m^3^ in the literature. Since the density of water is 1,000 kg/m^3^, the water carbon emission factor can be converted to 0.00091 kg CO_2_/kg.

#### 3.3.2. Materials CEF

*(1) Silicon-Containing Materials*. Sand and gravel are indispensable building materials for railway construction, but there are relatively few studies on carbon emissions during sand and gravel mining and processing. As the carbon emission measurement process for production and mining without sand and gravel in the reference, assuming that the measurement range is the same as this article, it can be directly quoted. The specific numerical calculations are shown in Table 4.

*(2) Blended Materials*. Since there is no carbon emission measurement process for bentonite, mineral powder, and fly ash in the references, assuming that the measurement range is the same as this article, it can be directly quoted, then the carbon of bentonite, mineral powder, and fly ash. The emission factors are 0.041 kg CO_2_/kg, 0.05692 kg CO_2_/kg, and 0.0015 kg CO_2_/kg.

*(3) Cement Materials*. The total carbon emission factor of cement can be obtained by summing the carbon emission factors of the raw material production stage, raw material transportation stage, and cement production and processing, as shown in Tables 3–8, that is, the cement carbon emission factors of PS32.5, PO42.5, and PI52.5 are, respectively, 802.259 kg CO_2_/t, 1,103.707 kg CO_2_/t, and 1,254.874 kg CO_2_/t.

*(4) Concrete Materials*. The production amount and processing energy consumption of different strength concrete raw materials are used to calculate the CEF in this study, namely C20, C25, C30, C35, C40, C50, and C60.

In the raw material production stage, five strength grades of concrete (C20, C25, C30, C35, and C40) use 42.5# cement, and two strength grades (C50 and C60) use 52.5# cement. The consumption of raw materials for concrete production is shown in Table 6.

The carbon emission factors of raw materials consumed in concrete production are shown in Table 7.

The carbon emission factors of the raw material production stage, the raw material transportation stage, and the concrete processing production stage are added together to obtain the concrete carbon emission factor, as shown in Table 8, that is, the carbon emission factors of the seven strength grades of concrete (C20–C60) are 306.192 kg CO_2_. /m^3^, 336.680 kg CO_2_/m^3^, 371.654 kg CO_2_/m^3^, 389.568 kg CO_2_/m^3^, 419.599 kg CO_2_/m^3^, 502.819 kg CO_2_/m^3^, and 549.342 kg CO_2_/m^3^.

*(5) Mortar Materials*. The carbon emission factor of cement mortar is obtained by adding the carbon emission factors of the raw material production phase, the raw material transportation phase, and the cement mortar processing production phase. As shown in Table 9, the carbon emission factors of the four different ratios of cement mortar are 829.388 kg CO_2_/m^3^, 636.038 kg CO_2_/m^3^, 581.347 kg CO_2_/m^3^, and 532.518 kg CO_2_/m^3^.

*(5) Steel Materials*. A large amount of steel is used in the railway construction stage, and the steel production stage consumes a lot of resources and energy to generate carbon emissions. Steel materials can be classified according to processes and uses, and there are large differences in the carbon emission factors of steel products of different uses and processes. Steel materials can be divided into screw steel, angle steel, section steel, round steel, and so on according to the purpose. As is presented in Table 10, the classification of steel in this study is that the four types of steel are large steel, medium and small steel, hot-rolled steel, and cold-rolled steel.

*(6) Wood Materials*. Timber is a commonly used turnover material for railway construction, such as wooden formwork, wooden support, and so on. This article believes that turnover wood is difficult to regenerate, that is, the turnover rate of turnover wood is 0. According to the above formula of turnover material carbon emission factor calculation formula, the turnover wood carbon emission factor can be obtained as 120.924 kg CO_2_/m^3^. Turnover timber amortization frequency is taken as 10 times, and its amortization uses CEF = 120.924/10 = 12.092 kg CO_2_/m^3^.  Table 11 presented the CEF of wood material.

The construction materials CEF of railway engineering are shown in Table 12.

#### 3.3.3. Facility CEF

The CEF of commonly used construction equipment for railway construction is shown in Table 13.

### 3.4. Measuring Model of the Carbon Emission

The carbon emissions from railway construction should include three aspects: carbon emissions from the transportation of building materials, carbon emissions from the use of building materials, and carbon emissions from construction. However, the use of construction machinery to assemble building materials does not directly generate carbon emissions. Carbon emissions related to building materials occur in the process of production, that is, carbon emissions from railway construction are “transferable.”

In this study, the production of building materials is listed separately before the construction phase, that is, it is divided into the building material production phase, the building material transportation phase, and the construction and construction phase. Based on the carbon emission measurement boundary, this research clarifies the content of carbon emission measurement at each stage and combs the carbon emission calculation formula.

(1) The calculation model of CEs during the production stage of building materials is shown in the following formula:
  (2) $$\begin{array}{c} C_{sc}=\sum_{i=1}^{n}m_{i}\times \left(1+U_{i}\right)\times C_{i}, \end{array}$$
where *C*_*sc*_ represents the carbon emissions during the production phase of building materials, *m*_*i*_ represents the consumption of building materials, *𝒰*_*i*_ denotes the building material loss rate, *c*_*i*_ represents the CEF of the building material production stage, and *n* represents the types of the building materials.
(2) The calculation model of CEs during the building materials transportation stage is shown in the following formula:.
  (3) $$\begin{array}{c} C_{ys}=\sum_{i=1}^{n}\sum_{j=1}^{k}m_{ij}\times \left(1+U_{i}\right)\times d_{ij}\times C_{i}, \end{array}$$
where *C*_*ys*_ represents the carbon emissions during the building materials transportation stage, *d*_*ij*_ denotes the average transportation distance of type *j* for construction materials (waste) *i*,*m*_*i*_ represents the consumption of building materials (amount of waste engineering), *𝒰*_*i*_ denotes the building material loss rate, and *c*_*i*_ represents the CEF of the building material production stage.
(3) The calculation model of CEs during the construction stage is shown in formula (4).
During the construction phase, carbon emissions are composed of two parts: the operation of construction machinery consumes energy (gasoline, diesel, electricity, etc.) to produce carbon emissions, the amortization of revolving materials produces carbon emissions, and the direct consumption of energy produces carbon emissions.
  (4) $$\begin{array}{c} C_{js}=C_{js1}+C_{js2}, \end{array}$$
where *C*_*js*_ represents the carbon emissions during the construction phase, *C*_*js*1_ denotes the construction machinery carbon emissions, *C*_*js*2_ represents the energy carbon emissions, *𝒰*_*i*_ denotes the building material loss rate, and *c*_*i*_ represents the CEF of the building material production stage.

The *C*_*js*1_ and *C*_*js*2_ can be obtained through the following equations:

(5) $$\begin{array}{c} C_{is1}=\sum_{l=1}^{a}h_{l}\times c_{l}=\sum_{m=1}^{b}r_{m}\times c_{m}, \end{array}$$

(6) $$\begin{array}{c} C_{is2}=\sum_{t=1}^{f}r_{t}\times c_{t}. \end{array}$$

## 4. Determining the Samples Implementing the MCDM

We collected 188 high-speed railway infrastructure construction projects in China using the average sampling method to complete the empirical research. These samples are China's important high-speed railway infrastructure construction projects. The Delphi method was used to determine whether these samples are resilient. MCDM selection techniques were used to determine the suitable MCDM methodology tailored to the decision process [79, 80]. The techniques adapted totally 9 alternatives for determining the required abilities from a set of 78 MCDM databases where the specific descriptors for the properties of the decision process are presented. For instance, qualitative, quantitative, and relative are regarded as the general standards for the alternative type of weights [81–83]. Finally, 26 samples are identified as resilient high-speed railway infrastructure construction projects.

The proposed measuring model was implemented to calculate the carbon emissions of the selected 26 projects.

## 5. Results and Discussions

We separately calculated the carbon emissions of these 26 resilient high-speed rail projects. Taking section A of the Huaihua-Hengyang (HH) high-speed railway project in China as an example, the measurement for the sample is adapted as follows.

The length of section A of the HH high-speed railway project is 66.95 km, including 44.36 km of tunnels, 9.65 km of bridges, and 12.94 km of roadbeds and stations; the proportion of bridges and tunnels is 80.7%; and the contract period is 60 months. The main project quantities are shown in Table 14.

1. The value of carbon emissions
2. The total carbon emission is calculated from the two dimensions of the construction stage and carbon emission source. The total carbon emission of materials is 1,253,677.42 t, of which the carbon emission in the production stage is 1,124,700.91 t and the carbon emission in the transportation stage is 128,976.52 t. The total carbon emission of construction equipment is 158,279.70 t. The total energy carbon emission is 7,167.56 t.
3. Comprehensive assessment of the carbon emissions
4. The results presented that the material production stage is the largest source of carbon emissions in the case of railway construction, accounting for 79%; the construction stage carbon emissions account for 12%; and the construction stage carbon emissions are the least, accounting for 9%. Moreover, the carbon emission contribution of materials is 88%; the carbon emission contribution of construction equipment is 11%; and the carbon emission of direct energy use only accounts for 1%. A comprehensive analysis of the data showed that reducing carbon emissions during material production is of great significance for controlling carbon emissions in high-speed railway construction.

The carbon emissions of cement and stone materials are higher than those of other building materials in the material production stage and material transportation stage. The high-speed railway construction in this study uses ready-mixed concrete. Cement, as the main building material for concrete production, consumes a huge amount of carbon, accounting for 54.38% and 25.83% of carbon emissions in production and transportation, respectively. As an important building material for concrete production, sand and gravel account for 16.80% of carbon emissions, second only to cement carbon emissions. The consumption of stone is smaller than that of cement, so the proportion of carbon emissions in the production process is lower than that of cement. However, due to the high density, a large amount of carbon emissions is generated in the transportation process. In summary, reducing carbon emissions from cement and sand production and transportation is the key to controlling carbon emissions from building materials.

Among the construction equipment, the top four contributors to carbon emissions are power machinery; transportation machinery; earth-rock machinery; foundation and pump machinery, with carbon emissions accounting for 37%, 26%, 17%, and 9%, respectively; hoisting machinery; and paving machinery. The carbon emissions from machinery, processing, and other machinery are relatively small. From this, it can be seen that the carbon emission reduction of construction equipment such as power machinery and transportation machinery with a large carbon emission contribution is the focus of carbon emission control of construction equipment.

Among the direct energy carbon emissions, electricity carbon emissions account for up to 73%, and water carbon emissions account for 26%. Direct consumption of fossil energy produces the least carbon emissions, accounting for only about 1%. Therefore, the energy and carbon emission reduction of construction sites can start by saving electricity and water resources.

After obtaining the carbon emissions of 26 resilient high-speed rail projects, we investigated the relationship between the resilience of the high-speed railway projects and the low-carbon emission. The results of the statistical analysis revealed that the resilience of the high-speed railway projects has a significant positive influence on low-carbon emissions.

## 6. Suggestions and Recommendations

### 6.1. Carbon Emission Control Strategy for the Government

Some scholars have called the climate change caused by excess carbon emissions, “the most serious and wide-ranging market failure in history,” and pointed out that only the coordinated efforts of the government and enterprises can avoid the irreversible consequences of excess carbon emissions. According to externality theory, effective government regulation can compensate for market failures. As a typical market failure, carbon emission requires effective government control to achieve its externality internalization. Based on literature research and domestic and foreign practice, it is concluded that carbon emission control strategies widely recognized at home and abroad mainly include carbon auditing, carbon tax collection, and carbon emission trading.

Railway construction carbon auditing refers to tracking and measuring the carbon emissions generated in the process of railway construction, reviewing the management of carbon emissions in the process of railway construction, and achieving the purpose of external intervention in carbon emissions. Carbon audit not only can realize the supervision of carbon emission reduction activities and promote the rational allocation of resources but also can contribute to the coordinated development of the economy and environment.

The participants in the carbon audit process of railway construction include the audit client, the carbon audit subject, and the carbon audit object. Among them, the principal-agent relationship between the audit client and the carbon audit object is the fundamental reason for carbon audit activities, and the audit content is the carbon emissions generated in the process of railway construction. The main body of carbon audit plays an important role in audit activities and can be divided into three categories: government audit subject, social audit subject, and internal audit. In the early stage of the development of carbon auditing in railway construction, China lacked relevant practical experience in carbon auditing in railway construction, and the audit risk was relatively high. Government auditing mainly assumed the main role of carbon auditing. Moreover, the government audit is highly authoritative, which is conducive to promoting the carbon audit of railway construction on the right track. With the gradual improvement of the carbon emission trading market, the participation of social audit subjects has gradually increased, which can play an important role in the carbon audit of railway construction. When the carbon emission trading market is relatively complete, the carbon emission audit of railway construction will become a routine audit business. At this time, the main body of internal audit was derived, and the role of carbon emission management in the process of railway construction was brought into full play.

Since it is currently impossible to implement mandatory carbon audits for all railway construction processes, this paper proposes the implementation framework of railway construction carbon audits concerning the “Kyoto Protocol.” Railway projects can be divided into three categories according to the priority of railway construction. The first category is the railway projects with mandatory carbon audit. The second category is the railway projects that are ready to implement carbon audit, and the third category is all the remaining railway projects. Then carbon audits are carried out for these three types of railway projects in three steps. Under the condition of gradual improvement, the implementation of carbon audits for the second type of railway projects has been promoted, and the construction of related systems such as carbon tax has been promoted. Furthermore, the carbon audit system is promoted in the construction process of all railway projects to achieve energy saving and emission reduction in the process of railway construction.

Based on the relevant economic theories, the negative external effects of carbon emissions originate from the coupling effect of government failure and market failure. To solve this problem, we must make full use of market instruments, which leads to carbon emission trading, a carbon emission response measure widely recognized and used by all countries in the world. The carbon audit of railway projects and the carbon emissions trading system promote and complement each other and can work together to help reduce carbon emissions. The attestation role of carbon audit can regulate market transactions and provide a basis of trust for both parties to the transaction. At the same time, carbon emission trading will also promote the development of carbon auditing, and the economic benefits brought by carbon emission trading will attract more carbon emission entities to participate. Finally, the market means to guide the construction unit's carbon audit activities.

To ensure the sustainable, long-term, and healthy development of the carbon audit system for railway projects, we should also build a friendly audit environment for carbon audit of railway projects from the perspectives of politics, economy, law, and social environment.

The economic principle of carbon emission trading involves three classic theories of resource scarcity, externality, and property rights. The theory of resource scarcity reveals the deep root of carbon emissions trading. The negative externality of carbon emissions is the direct cause of emissions trading, and the definition and trading of carbon emissions provide solutions for the internalization of negative externalities of carbon emissions. According to economic theory, carbon emission behaviors enter the market without clear property rights, resulting in significant negative external effects. Economists believe that based on the initial allocation of carbon emissions within the quota, carbon emission rights can be regarded as a tradable commodity and allowed to circulate freely, to achieve the purpose of controlling carbon emissions and achieving economic benefits. In the exploration of carbon emission rights trading in the past 10 years, China has laid a solid foundation for the construction of a unified national carbon emission rights trading market and has also contributed to the early establishment of a carbon emission rights trading system. This study explores key regimes for rail carbon emissions trading.

Government regulation can be divided into two stages: carbon emission reduction regulation and carbon emissions trading regulation, which are implemented through the following mechanisms. The first is the quota allocation supervision mechanism. Whether the allocation of carbon emission allowances is fair and effective is directly related to the normal operation of the carbon emission trading market. The competent department of carbon emission allowance allocation should set up a reasonable and effective supervision system and take measures such as introducing a notary public for supervision and implementing allowance allocation through an online carbon emission allowance allocation system to ensure fair distribution. The second is the regulatory mechanism for trading market behavior. The government should supervise the carbon emission trading process strongly to ensure the trading order. On the one hand, qualification checks can be set up. The carbon emission rights exchange should conduct qualification examinations on carbon emission rights trading entities and set membership criteria. Only those who meet the standards can join the membership. On the other hand, transaction monitoring is possible. Exchanges can establish a transaction monitoring platform to monitor transaction information in real time. The third is the performance offset supervision mechanism. Carbon emission compliance and write-off directly affect the emission reduction results of railway projects, so they must be taken seriously. The carbon emission rights trading authority should formulate a time scale for compliance and urge emission reduction units to submit carbon emission quotas promptly. Competent authorities should also focus on carbon emissions trading volumes in carbon emissions trading and conduct data verification. After the implementation of the contract, the competent department should cancel the quota that has been implemented in time to lay the foundation for the next round of carbon emission reduction implementation.

In addition to supervision, the carbon emission rights trading of railway projects should also set up a penalty mechanism to achieve constraints on emission reduction units. The punishment mechanism should not only punish those who fail to meet the emission reduction targets but also cannot affect the enthusiasm of carbon emission entities to participate in carbon emission trading. In practice, a combination of various punishment methods can be considered.

The first is to set up a mechanism for the disclosure of energy efficiency of railway projects. The key to carbon emission trading of railway projects is the lack of accurate energy consumption and carbon emission data. At present, the energy consumption data of railway projects are not public, which is not conducive to the promotion of carbon emission reduction of railway projects. China can learn from the practical experience of developed countries, set up a special carbon emission information disclosure agency, and require enterprises to include emission reduction information in their annual reports to facilitate supervision by the competent authorities. The second is to set up an overquota price increase mechanism. For small projects, when the carbon emission exceeds the allocated carbon emission quota, the overquota price increase system can be adopted concerning the electricity price. This kind of pricing utilizes a progressive price lever, which is conducive to guiding emission reduction entities to conduct spontaneous emission reductions. In the specific implementation process, relevant departments need to coordinate and cooperate to jointly determine the data such as the price increase rate.

The incentive system is the opposite of the penalty system, and positive incentives are used to promote the development of the carbon emissions trading market. In the early stage of the establishment of the market, the relevant system is not perfect, and the participants are limited. The role of the incentive system should be brought into full play to encourage carbon emission entities to actively participate in carbon emission trading so that the role of the carbon emission trading market can be brought into full play.

On the one hand, it can make full use of market adjustment funds. In the early stage of the establishment of the carbon emission rights market, a unified national normative system has not yet been established, and the participation of carbon emission entities is less, resulting in a shortage of demand. The government should play a role at this time to stimulate the demand for carbon emissions trading, allocate funds to set up special funds, and stimulate market vitality. When the market develops gradually, the government can buy or sell the carbon emission allowances it holds according to the actual market conditions, to achieve the purpose of market regulation. After the market matures, it is no longer necessary for the government to fully invest in the establishment of special funds, which can be composed of various sources such as fines for violations and social donations, to achieve the sustainability of funds. On the other hand, support should be provided for railway energy-saving technologies. The carbon emission of railways is relatively large, and the realization of carbon emission reduction requires long-term continuous promotion, and the key to realizing carbon emission reduction is the research and development and promotion of energy-saving technologies. The government should fully support the technical needs of emission reduction entities, carry out research on energy conservation and emission reduction in relevant national or local research centers, increase financial support, and vigorously promote low-carbon railway technology research and railway low-carbon equipment upgrades.

### 6.2. Carbon Emission Control Strategies of Construction Enterprises

The carbon emission control strategies of construction enterprises focus on low-carbon materials, environmental protection construction techniques, and clean energy. The carbon emission information integrated management platform and various information tools can effectively help reduce carbon emissions. As an important participant in railway engineering construction and the main promoter of carbon emission reduction in railway construction, the construction unit should implement the concept of low-carbon construction and optimize on-site management; it can also make full use of information tools such as BIM to achieve integrated management of railway carbon emissions information.

Due to the huge volume of railway projects, carbon emission measurement needs to call a large amount of engineering data. Manually exporting engineering quantities and then performing carbon emission measurement is time-consuming and inefficient, and carbon emission measurement cannot be correlated with information such as construction progress and cost. BIM technology can meet the above requirements at the same time. Therefore, a BIM model of railway engineering construction should be constructed to integrate various information such as railway construction project quantity, progress, cost, and carbon emissions to provide information technology support for railway carbon emissions management.

The integrated management of carbon emission information in railway engineering construction refers to the combination of low-carbon information in the railway engineering construction stage and the BIM model to build a low-carbon information database in the railway engineering construction stage and at the same time integrate construction data (construction progress, railway cost, etc.) with low-carbon information, realize the real-time measurement of carbon emissions in the construction phase of railway projects, and analyze the influencing factors of carbon emissions accordingly. Its essence is to add progress information, cost information, and carbon emission information based on the 3D BIM model to build a 6D BIM model. The carbon emission information integrated management model can realize the carbon emission management in the construction process. By monitoring the progress, cost, carbon emission, and other data displayed in the model in real-time, the influencing factors of carbon emission in the construction process can be analyzed, which can provide a reference for the selection of schemes and promote railway construction carbon emission management.

The implementation steps of the railway carbon emission integrated management model are as follows: first, collect carbon emission data. Carbon emission data are the prerequisites for the integrated management of carbon emission information in the construction phase of railway projects, including railway engineering volume data and carbon emission factor data. The railway engineering quantity data can be obtained directly from the railway BIM model, and the carbon emission factor can be queried in the authoritative carbon emission factor database. Second, integrate schedule data, cost data, and carbon emissions data in the BIM model. The construction progress plan is imported into the BIM model as construction progress information, and the on-site construction progress of the railway construction stage is controlled in real-time; the price information of different regions has been included in the BIM software, and the bill of quantities can be coded to summarize the railway construction cost data. The carbon emission data of the BIM model is added to the BIM model as a resource, and the carbon emission generation process is regarded as the resource consumption process, and the resource consumption curve diagram of the construction schedule is obtained.

## 7. Conclusion

We collected 188 high-speed railway infrastructure construction projects in China using the average sampling method to complete the empirical research. These samples are China's important high-speed railway infrastructure construction projects. The Delphi method was used to determine whether these samples are resilient. Finally, 26 samples are identified as resilient high-speed railway infrastructure construction projects.

The proposed measuring model was implemented to calculate the carbon emissions of the selected 26 projects. Achieving a resilient transport infrastructure is imperative to building a modern society. At the same time, the resilient transport infrastructure requires a combination and investment of multiple resources that have caused concern about the carbon emissions of resilient transportation infrastructure. Therefore, from this perspective, this study developed a carbon emission measurement framework for evaluating the carbon emission of several selected resilient transport infrastructure projects. Twenty-six samples are finally identified as resilient high-speed railway infrastructure construction projects. The results revealed a relatively high carbon emission in these resilient high-speed railway infrastructure construction projects. Resilient transport infrastructure with lower carbon emissions is located in remote cities.

The findings could help investigate the carbon emission of resilient transport infrastructure projects. The correlation between resilience and carbon emission is useful for policy-makers to conduct an effective plan for the cities.

## Figures and Tables

**Table 1:** Carbon emission factor from the literature.

Factor	Unit	CEF	Production processes						
			Fossil energy mining	Raw material acquisition	Raw material transportation	Processed into lumber	Building materials transportation	Regeneration treatment	Source of data
Sand	m^3^	72.5		✓	✓	✓			[48]
Stone	m^3^	31.2		✓	✓	✓			[49]
Fly ash	kg	0.0015		✓	✓	✓			[50]
Bentonite	kg	0.041		✓	✓	✓			[51]
Mineral powder	kg	0.05692		✓	✓	✓			[52]
32.5#cement	t	677.68	✓	✓	✓	✓			[52]
42.5# cement	t	920.03	✓	✓	✓	✓			[53]
52.5# cement	t	1,041.56	✓	✓	✓	✓			[54]
C20 concrete	m^3^	239.19		✓	✓	✓	✓		[55]
C25 concrete	m^3^	289.44		✓	✓	✓	✓		[56]
C30 concrete	m^3^	346.95		✓	✓	✓	✓		[57]
C35 concrete	m^3^	382.11		✓	✓	✓	✓		[58]
C40 concrete	m^3^	432.29		✓	✓	✓	✓		[59]
C50 concrete	m^3^	563.89		✓	✓	✓	✓		[60]
C60 concrete	m^3^	644.85		✓	✓	✓	✓		[61]
1:1 cement mortar	m^3^	730.20		✓	✓	✓			[62]
1:2 cement mortar	m^3^	531.52		✓	✓	✓			[63]
1:2.5 cement mortar	m^3^	469.41		✓	✓	✓			[64]
1:3 cement mortar	m^3^	393.65		✓	✓	✓			[65]
Large steel	kg	1.72		✓	✓	✓		✓	[66]
Small and medium steel	kg	1.38		✓	✓	✓		✓	[67]
Hot rolled steel bar	kg	2.21		✓	✓	✓		✓	[68]
Cold rolled steel bar	kg	2.76		✓	✓	✓		✓	[69]
Iron product	kg	1.53		✓	✓	✓		✓	[70]
Wood	m^3^	144.5		✓	✓	✓			[71]
Waterproof coating	kg	1.21	✓	✓	✓	✓	✓		[72]
		1.01	✓	✓	✓	✓			[73]
		0.89		✓	✓	✓			[74]
Modified asphalt waterproof materials	m^2^	4.28	✓	✓	✓	✓	✓		[75]
		4.01	✓	✓	✓	✓			[76]
PVC waterproof board	kg	8.69		✓	✓	✓			[77]
Rubber waterstop	kg	0.5		✓	✓	✓			[78]

**Table 2:** Fossil energy CEF.

Fossil energy	Net calorific value	Carbon content	Carbon dioxide factor (%)	Unit	CEF
Raw coal	20,908	25.8	100	kg	1.978
Washed coal	26,344	25.8	100	kg	2.492
Coke	28,435	29.2	100	kg	3.044
Crude	41,816	20.0	100	kg	3.067
Kerosene	43,070	19.5	100	kg	3.080
Gasoline	43,070	18.9	100	kg	2.985
Diesel fuel	42,652	20.2	100	kg	3.159
Liquefied petroleum gas	50,179	17.2	100	kg	3.165
Natural gas	38,931	15.3	100	m^3^	1.996
Coke oven gas	16,726	12.1	100	m^3^	0.770

**Table 3:** Fossil energy CEF.

Region	OM electricity CEF	BM electricity CEF
North China power grid	0.9419	0.4819
Northeast power grid	1.0826	0.2399
Northwest power grid	0.8922	0.4407
East China power grid	0.7921	0.3870
Central China power grid	0.8587	0.2854
China southern power grid	0.8042	0.2135

**Table 4:** Silicon-containing materials CEF.

Silicon-containing materials	Bulk density (kg/m^3^)	CEF (kg CO_2_/m^3^)	CEF (kg CO_2_/kg)
Stone	1,560	31.2	0.02
Sand	1,450	72.5	0.05

**Table 5:** Cement materials CEF.

CEF	Raw material production stage	Raw material transportation stage	Cement production and processing stage	Total
P.S.32.5	517.100	40.498	244.661	802.259
P.O.42.5	729.200	44.211	330.296	1,103.707
P.I.52.5	835.550	46.092	373.232	1,254.874

**Table 6:** Consumption of raw materials for concrete production.

Materials	C20	C25	C30	C35	C40	C50	C60
Cement	135	170	210	235	270	320	370
Fly ash	70	70	70	75	80	80	80
Mineral powder	80	80	80	80	80	80	90
Sand	843	825	805	755	732	723	682
Stone	1,020	1,020	1,020	1,020	1,020	1,025	1,000
Water	185	185	180	180	180	165	170
Admixture	1.18	1.38	3.64	4.1	4.9	7	8.3

**Table 7:** Concrete raw material CEF.

Raw materials	42.5# cement	52.5# cement	Admixture	Stone	Sand	Water	Mineral powder	Fly ash
CEF	1.104	1.255	0.02849	0.02	0.05	0.00091	0.05692	0.0015

**Table 8:** Concrete material CEF.

CEF	C20	C25	C30	C35	C40	C50	C60
Raw material production	184.051	213.396	247.016	266.137	295.257	375.593	422.704
Raw material transportation stage	119.431	120.574	121.928	120.721	121.632	124.516	123.928
Concrete production and processing stage	2.710154	2.710154	2.710154	2.710154	2.710154	2.710154	2.710154
Total	306.192	336.680	371.654	389.568	419.599	502.819	549.342

**Table 9:** Concrete material CEF.

CEF	1:1 cement mortar	1:2 cement mortar	1:2.5 cement mortar	1:3 cement mortar
Raw material production	712.694	514.127	457.936	409.636
Raw material transportation stage	115.086	120.303	121.803	121.274
Mortar production and processing stage	1.608	1.608	1.608	1.608
Total	829.388	636.038	581.347	532.518

**Table 10:** Steel material CEF.

Steel type	CEF	Categories
Large steel	3,612.011	Section steel, I-beam
Small and medium steel	2,895.229	Channel steel, angle steel, steel plate, steel support, steel formwork, steel support
Hot rolled steel bar	3,041.139	Rebar, round steel
Cold rolled steel bar	3,786.384	Cold drawn steel wire

**Table 11:** Wood material CEF.

Production process	Log harvesting	Log transportation	Timber processing
Energy	Gasoline	Diesel fuel	Electricity
Number	16.487 (kg/m^3^)	4.844 (kg/m^3^)	70.142 (kWh/m^3^)
CEF (kg/CO_2_)	2.985	3.159	0.8042
CEF (m^3^/CO_2_)	49.214	15.302	56.408

**Table 12:** Construction materials CEF of the high-speed railway project.

Types	Materials	Unit	CEF
Nonturnover material	Stone	m^3^	31.2
	Sand	m^3^	72.5
	Bentonite	kg	0.041
	Mineral powder	kg	0.05692
	Fly ash	kg	0.0015
	32.5#cement	t	802.259
	42.5# cement	t	1,103.707
	52.5# cement	t	1,254.874
	C20 concrete	m^3^	306.192
	C25 concrete	m^3^	336.680
	C30 concrete	m^3^	371.654
	C35 concrete	m^3^	389.568
	C40 concrete	m^3^	419.599
	C50 concrete	m^3^	502.819
	C60 concrete	m^3^	549.342
	1:1 cement mortar	m^3^	829.388
	1:2 cement mortar	m^3^	636.038
	1:2.5 cement mortar	m^3^	581.347
	1:3 cement mortar	m^3^	532.518
	Large steel	t	3,612.011
	Small and medium steel	t	2,895.229
	Hot rolled steel bar	t	3,041.139
	Cold rolled steel bar	t	3,786.384
	Iron product	t	2,084.565
	Wood	m^3^	120.924
	Waterproof coating	kg	0.89
	Modified asphalt	m^2^	3.53
	Waterproof materials	m^2^	19.553
	PVC waterproof board	m	4.608
Reusable materials	Rubber water stop	t	1,331.805
	Turnover steel	m^3^	12.092

**Table 13:** Facility CEF of the high-speed railway project.

Types	Construction equipment	Energy consumption			CEF
		Gasoline (kg)	Diesel fuel (kg)	Electricity (kWh)	
Earthwork machinery	Crawler hydraulic single bucket excavator ≤0.4 m^3^	—	35.48	—	112.08
	Crawler hydraulic single bucket excavator ≤0.6 m^3^	—	44.08	—	139.25
	Crawler hydraulic single bucket excavator ≤1 m^3^	—	62.90	—	198.70
	Crawler bulldozer ≤75 kW	—	49.73	—	157.10
	Crawler bulldozer ≤300 kW	—	197.57	—	624.12
	Self-propelled vibratory roller ≤12 t	—	75.00	—	236.93
	Frog ram ≤700 Nm	—	—	20.40	16.41
	Wheel loader ≤2 m^3^	—	56.45	—	178.33

Lifting machinery	Truck crane ≤8 t	—	35.28	—	111.45
	Truck crane ≤16 t	—	57.15	—	180.54
	Gantry crane ≤10 t–22 m	—	—	61.44	49.41
	Gantry crane ≤20 t–22 m	—	—	109.44	88.01
	Gantry crane ≤50 t–40 m	—	—	176.64	142.05
	Crawler crane ≤10 t	—	31.75	—	100.30
	Crawler crane ≤15 t	—	38.81	—	122.60
	Crawler crane ≤40 t	—	47.63	—	150.46
	Crawler crane ≤250 t	—	352.80	—	1,114.50
	Single drum slow speed winch ≤30 kN	—	—	38.40	30.88
	Single drum slow speed winch ≤50 kN	—	—	56.32	45.29

Transportation machinery	Dump truck ≤4 t	—	34.27	—	108.26
	Dump truck ≤8 t	—	47.58	—	150.31
	Dump truck ≤12 t	—	61.29	—	193.62
	Truck ≤4 t	26.61	—	—	79.43
	Truck ≤6 t	34.56	—	—	103.16
	Sprinkler ≤5,000 L	34.56	—	—	103.16
	Small transport vehicle ≤1 t	—	7.26	—	22.93
	Belt conveyor ≤10 m	—	—	15.36	12.35
	Concrete mixing truck ≤6 m^3^	—	88.70	—	280.20
	Concrete mixing truck ≤8 m^3^	—	100.80	—	318.43
	Concrete mixing truck ≤10 m^3^	—	106.85	—	337.54

Concrete and mortar machinery	Concrete mixer ≤250 L	—	—	15.68	12.61
	Concrete mixer ≤400 L	—	—	21.56	17.34
	Concrete mixer ≤800 L	—	—	86.24	69.35
	Concrete mixing station ≤60 m^3^/h	—	—	636.16	511.60
	Concrete mixing station ≤100 m^3^/h	—	—	913.92	734.97
	Concrete mixing station ≤120 m^3^/h	—	—	1,008.00	810.63
	Concrete plug-in vibrator	—	—	5.38	4.33
	Concrete attached vibrator	—	—	6.72	5.40
	Suspended pulp lifting and leveling machine	—	—	105.28	84.67
	Concrete wet spraying machine ≤5 m^3^/h	—	—	24.64	19.82
	Hydraulic grouting pump ≤50 L/min	—	—	30.80	24.77
	Concrete pump ≤60 m^3^/h	—	—	492.80	396.31
	Concrete pump truck ≤90 m^3^/h	—	61.74	—	195.04
	Concrete placing machine ≤21 m	—	—	21.84	17.56
	Mortar mixer ≤200 L	—	—	13.44	10.81
	Mortar mixer ≤400 L	—	—	20.16	16.21
	Prestressed steel bar hydraulic tensioning equipment ≤1,200 kN	—	—	38.40	30.88
Foundation and pump machinery	Hydraulic vibration pile driver ≤320 t	—	650.92	—	2,056.26
	Hydraulic static pile driver ≤1,200 kN	—	—	138.60	111.46
	Hydraulic static pile driver ≤1,600 kN	—	—	189.00	151.99
	Impact hole forming machine *d* ≤ 1.5 m	—	—	177.60	142.83
	Crawler hydraulic grab grooving machine ≤1.2 m	—	194.04	—	612.97
	Dynamic compaction machinery ≤1,200 kNm	—	56.70	—	179.12
	Dynamic compaction machinery ≤2,000 kNm	—	69.30	—	218.92
	Single-stage centrifugal clean water pump ≤12.5 m^3^/h–20 m	—	—	8.98	7.22
	Single-stage centrifugal clean water pump ≤50 m^3^/h–38 m	—	—	44.88	36.09
	Multi-stage centrifugal clean water pump ≤85m³/h–180m	—	—	224.40	180.46
	Multi-stage centrifugal clean water pump ≤155 m^3^/h–185 m	—	—	538.56	433.11
	Sewage pump ≤90 m^3^/h–26 m	—	—	89.76	72.18
	Centrifugal mud pump ≤108 m^3^/h–21 m	—	—	89.76	72.18
	Mud water treatment centrifuge ≤100 m^3^/h	—	—	326.40	262.49
	Mud water separation equipment ≤1,500 m^3^/h	—	—	1,836.00	1,476.51
	Mud production cycle equipment ≤500 m^3^/h	—	—	136.00	109.37

Welding machinery	AC arc welding machine ≤42 kVA	—	—	144.00	115.80
	DC arc welding machine ≤32 kW	—	—	102.40	82.35
	Butt welding machine ≤100 kVA	—	—	288.00	231.61

Pavement machinery	Track laying machine 25 m	—	193.64	—	611.71
	Long rail laying unit for ballastless track 500 m	—	94.25	—	297.74
	Turnout tamping car	—	298.17	—	941.92
	Long rail line laying and rolling mill	—	182.50	—	576.52
	Bridge erecting machine ≤900 t	—	642.03	—	2,028.17
	Box beam transport vehicle ≤900 t	—	913.92	—	2,887.07
	Wheel-rail beam moving machine ≤900 t	—	188.50	—	595.47
	Wheel rail type beam lifting machine ≤2 × 450 t	—	188.50	—	595.47
	Rail slab reinforcement tensioning equipment	—	—	105.60	84.92
	Type I double-block sleeper concrete pouring production line	—	—	384.00	308.81

Processing and other machinery	Steel bar straightening machine, *d* ≤ 14	—	—	18.70	15.04
	Rebar cutting machine, *d* ≤ 40	—	—	33.32	26.80
	Rebar bending machine, *d* ≤ 40	—	—	14.28	11.48
	Woodworking circular saw machine, *d* ≤ 500	—	—	16.32	13.12
	Jaw crusher, ≤250 × 400	—	—	81.60	65.62
	Vertical drilling machine, *d* ≤ 25	—	—	8.98	7.22
	Pipe cutting machine, *d* ≤ 150	—	—	13.60	10.94

**Table 14:** Categories of subprojects of section A of the HH project.

No.	Categories	Projects	Numbers
1	Earthworks	Subgrades	1.69 million m^3^
2		Stations	2.2 million m^3^
3	Bridges	Mega bridge	3,517 m
4		Large bridge	5,580 m
5		Middle bridge	557 m
6		Small bridge	49 m
7		Culverts	1,638 m
8	Tunnels		44,057 m
9	Buildings		14,404 m^2^

## Data Availability

All data sets generated for this study are included in the article.
